# Heavy metal removal from MSS fly ash by thermal and chlorination treatments

This article has been retracted.

**DOI:** 10.1038/srep17270

**Published:** 2015-11-25

**Authors:** Jingyong Liu, Jiacong Chen, Limao Huang

**Affiliations:** 1 School of Environmental Science and Engineering, Guangdong University of Technology, Guangzhou 510006, China

## Abstract

The thermal behavior of heavy metals in the co-incineration of municipal solid waste-sludge incinerator fly ash (MSS fly ash) was studied using a laboratory-scale tube furnace. The results indicate that without the addition of chlorinating agents, temperature was an important parameter and had significantly influenced on heavy metal removal, whereas the residence time had a weak effect. Between 900 and 1000 °C for 60 to 300 min, heavy metals reacted with chloride-inherent in the fly ash, and approximately 80 to 89% of Pb, 48% to 56% of Cd, 27% to 36% of Zn and 6% to 24% of Cu were removed. After the adding chlorinating agents, the evaporation rate of the heavy metals improved dramatically, where the evaporation rates of Cu and Zn were larger than that of Pb and Cd. As the amount of added chlorinating agents increased, the removal rate of heavy metals increased. However, the effect of the type of chlorinating agent on the chlorination of heavy metals differed considerably, where NaCl had the weakest effect on the removal rate of Cu, Cd and Zn. In terms of resource recovery and decontamination, MgCl_2_ and CaCl_2_ are the best choices due to their efficient removal of Zn.

The production of sewage sludge is rapidly increasing, and its treatment has attract considerable attention in recent years^1^. Compared with landfill and agricultural use, incineration is preferred for quick disposal, large volume and weight reduction ratio and energy recovery^2^. In China, the co-combustion of sludge and municipal solid waste (MSW) or coal for power generation is becoming the primary method of sludge incineration due to the number of available incineration plants with advanced equipment^3^. However, during this process, the amount of incineration residues produced, which include bottom ash and fly ash, can reach 10 wt.% of the total mass of feedstock and contains large amounts of heavy metals^4^.

There are many patented processes concerning the disposal or usage of these incineration residues, particularly for fly ash disposal. These processes can be classified as follows^5^: (1) fly ash mixed with a binder (e.g., inertization in a cement matrix); (2) fly ash treated hydrometallurgically for heavy metal removal and (3) fly ash treated thermally with the objective of inertization and/or heavy metal removal (e.g., melting or sintering). However, many of these processes have disadvantages. Using the first method as an example, once fly ash is hardened in a cement matrix, the heavy metals are diluted. Hence, it is more difficult and costly to recover metals at a later stage. Additionally, the binding of heavy metals (hydraulically in a cement matrix or after melting as glass) does not mean complete immobilization^6^. Thus, heavy metal separation from fly ash is becoming important as a source for metal recovery or as a means to reduce its potential hazards.

A process that would remove heavy metals prior to landfill disposal is desirable^7^,^8^,^9^, particularly if this process could simultaneously recover contaminant heavy metals. A dry process, such as a thermal treatment, is potentially attractive, which could separate certain heavy metals from the bulk matrix (SiO_2_, Al_2_O_3_ and CaO) of the ash by forming metal chlorides at lower temperatures^10^. Thermal treatment of fly ash causes both the evaporation and stabilization of heavy metals depending on the treatment temperature^11^,^12^. Jakob *et al.* found that the evaporation of Zn, Pb, Cd and Cu in an electrostatic precipitator ash was most effective at temperatures just below the melting range of the ash (1000–1100 °C)^11^. However, the treatment types of ash melting require high energy consumption and produce secondary fly ash^13^. Heavy metal chlorides generally have high vapor pressures and lower boiling points compared with those of the corresponding metal oxides^14^. The condensation process of these metal compounds can be delayed when Cl is involved during thermal treatment, which can accelerate the volatilization of heavy metals. Thus, MSS fly ash could be mixed with a certain quantity of chlorinating agents to effectively separate heavy metals from MSS fly ash^15^,^16^. For industrial application, solid chlorinating agents (e.g., NaCl, MgCl_2_ or CaCl_2_) are advantageous because of (1) the simpler handling compared with gaseous Cl_2_, and (2) the fact that Cl_2_ also leads to the chlorination of non-hazardous elements, such as Ca or Fe (i.e., CaCl_2_, which has been used in a previous study in addition to Cl_2_, is more selective for Cd, Cu, Pb and Zn)^17^,^18^,^19^,^20^.

For example, Chan *et al.* reported that the chlorinating agents CaCl_2_ and Cl_2_ have significant influence on the volatilization of heavy metals in fly ash^20^. Nowak *et al.* found that more than 90% of Cd and Pb, nearly 60% of Cu and 80% of Zn could be removed from MSW fly ash by mixing with CaCl_2_^5^. During these processes, certain heavy metals will still volatilize and discharge, which will not only increase the burden on subsequent flue gas treatment systems but will also cause secondary pollution^21^,^22^,^23^,^24^. Previous research on heavy metals in solid waste incineration ash has generally focused on solidification and stabilization. Thermal separation technology of heavy metals primarily exists for MSWI fly ash but is less common for MSS fly ash. In fact, the matrix composition of MSS fly ash is a significantly different from that of pure MSWI ash. Previous studies have shown that the volatilization of heavy metals is related to their matrix, physical/chemical properties and the operation conditions^25^,^26^. Therefore, before conducting thermal treatment or recovery of the heavy metals in MSS fly ash, it is necessary to investigate and identify the factors that affect affecting the transformation and volatilization of heavy metals.

The objective of this study was to identify the conditions under which heavy metals would be effectively removed by adding various chlorinating agents. The parameters investigated in this study were the heating temperatures, heating time and types and amounts of chlorinating agents (CaCl_2_, MgCl_2,_ NaCl, FeCl_3_ and AlCl_3_). The feasibility of using a single heating process to remove heavy metals from fly ash was evaluated. The results improve our basic understanding of the underlying processes of heavy metal release from MSS fly ash and provide a theoretical basis for the highly efficient and harmless recovery of heavy metals from MSS fly ash.

## Method section

### Samples and reagents

The MSS fly ash was taken from a waste-to-energy (WTE) plant (co-incineration of MSW and semi-dry sewage sludge) from the Zhejiang Province, China. The raw feedstock included MSW and sewage sludge, in which the weight of the sewage sludge was approximately 50%. The plant contains three parallel industrial waste incinerator lines and has a treatment capacity of 3 × 500 t/d. The flue gas is cleaned by bag filter combined with the semi-dry method. The fly ash samples are mixtures of ashes from two incineration lines, which are collected in the vessels and the bag filters. The samples were passed through a 20-mesh sieve and were well mixed by a tumbling mixer in the laboratory. Before thermal treatment experiments, the ash samples were dried at 105 °C for 24 h.

The chlorinating agents used were NaCl, FeCl_3_·6H_2_O, MgCl_2_·6H_2_O, AlCl_3_ and CaCl_2_. NaCl is grained similar to that of common salt, and MgCl_2_ and CaCl_2_ are in flake form. Additionally, CaCl_2_ was ground in a ball mill before the experiment. All of the chemicals used were of analytical grade (AR). The amounts of chlorinating agents were used as-received based on the chlorine (Cl) content. Amounts of 0, 10, 50, 150 and 200 g Cl/kg ash was added to the MSS fly ash. The MSS fly ash and chlorinating agents were mixed and homogenized before conducting the experiments.

### Experimental apparatus

As shown in Fig. 1, the apparatus used in this study consisted of an air supply device, an electric-heated tube furnace and smoke absorber. The incineration chamber was a 60-mm long quartz tube with an inner diameter of ¢ = 20 mm. The chamber used a SK2-2-130 fast heating-up tube furnace with a PID self-tuning function (manufactured by Tianjin Zhonghuan Laboratory Electric Stove Co., Ltd.), and its temperature tracking precision was ±2 °C. A quartz tube burner was placed in a glass fiber-lined-insulated steel shell, and a quartz boat, which could be moved by a quartz rod, was used to feed the MSS fly ash into the furnace tube. The tube furnace, which was the main body of the setup, was a high alumina furnace tube surrounded by external heating wires. The combustion temperature at the center inside the furnace tube was monitored by a thermocouple and controlled by a programmable temperature controller. The furnace tube was horizontally placed to provide a stable temperature that could be set between 0–1200 °C as needed. The temperature control system had two modes, i.e., the KSY series control used intelligent temperature control instruments and special modules with high control precision and over-temperature protection.

### Experimental procedure

Samples of fly ash and different types of chlorinating agents were accurately weighed. The chlorinating agents, which were in powder form, were thoroughly mixed homogeneously with the ash in a weighing dish using a glass stirring rod before being transferred to the alumina boat. During heating, dry air was supplied at approximately 120 mL/min to entrain the volatile matter combustion. On leaving the end of the furnace, the volatile matter first condensed partially on the wall of the quartz tube outside the heating zone and then on the condensation tube. The outlet gases flowed through two absorption bottles filled with a 5% (*v/v*) HNO_3_ solution to clean the volatile components. Once the furnace temperature reached the target value, a porcelain boat filled with a 5 g fly ash sample was slowly pushed into the furnace. Then, the carrier gas was adjusted to the set value, and the furnace door was closed. After a certain residence time, the porcelain boat was removed and cooled to room temperature. Then, the residue slag at the bottom of the porcelain boat was collected for heavy metal detection. For the pure MSS fly ash, experiments were performed at 900 and 1000 °C and at a residence time of 1, 1.5, 2, 3, 4 and 5 h under the same thermal conditions mentioned above. To determine the repeatability and consistency of the results, each experiment was repeated three times.

Previous studies have proven that this experimental tube furnace can effectively simulate the volatilization of heavy metals during a high-temperature treatment^16^,^27^,^28^. In this experiment, the heavy metal compounds that evaporated from the fly ash were mostly absorbed by the absorption solutions, and only a small amount adhered to the internal surface of the quartz tube (around the outlet area) and inner wall of the catheter. To enhance the test accuracy, the quartz tube and catheter should be cleaned by a small amount of solution after each experiment.

To quantify the volatility of the heavy metals Cu, Pb, Zn and Cd, the efficiency volatilization *Ψ*/% is used, which is defined as the percentage of a metal that is removed from the MSS fly ash. *Ψ* is defined by equation (1)^29^,^30^:



where *Ψ* is the volatilization rate (%), *c*_1_ is the element content in the untreated sample (mg/kg), *m*_1_ is the mass of the untreated sample (g), *c*_2_ is the element content in the treated sample (mg/kg), and *m*_2_ is the mass of the treated sample (g).

### Analysis method

The original fly ash and heat-treated residues were milled and screened by a 150-mesh sieve. The major element compositions were measured by X-ray fluorescence (XRF) spectrometry (Rigaku 100e) on fused glass disks following the previous analytical procedures^31^, and where analytical precision for major elements was between 1 and 5%.

The heat-treated and untreated samples were dried, pulverized, completely digested with a mixture of HNO_3_, HF and HClO_4_ and analyzed with FAAS for Cd, Pb, Cu and Zn following the USEPA3050 method. All determinations were performed by triplicate, and differences between replications were less than 6%. The average value was calculated, and the relative standard deviations (RSD) for Cd, Pb, Cu and Zn were 3.2, 2.4, 2.7 and 1.6%, respectively.

The sample composition was analyzed by X-ray fluorescence (XRF) (Bruker RS 3000, Be source, Rh-anti-cathode, OVO 55 analyzer crystal) using a standard-less method (semi-quantitative analysis) and Spectra Plus software. All possible crystalline phases and metal speciation in the pure and chlorinated fly ash (milled) were investigated by a Rigaku DPmax2400 X-ray diffractometer (XRD) using a PANalytical X’Pert PRO powder diffractometer with a Cu(LFF) anode (λ(K_α1_) = 1.5406 Ǻ, λ(K_α2_) = 1.5444 Ǻ; 40 kV, 40 mA) and an X′Celerator detector (Ni K_β_ filter). Scans were recorded in the region 2θ = 10–90° within a measuring time of 14 min. For qualitative and quantitative interpretation, the databases Powder Diffraction File (PDF; International Centre for Diffraction Data ICDD, Newtown Square, PA/USA, 2001) and the Inorganic Crystal Structure Database (ICSD, Karlsruhe/Germany, 2007), were used, respectively. The morphological characteristics of selected bottom ash samples were also examined using a scanning electron microscope (SEM), and qualitative elemental analysis was conducted using energy dispersive X-ray spectroscopy (EDS) (S-3400N-II, Hitachi, Japan).

## Results and Discussion

### Physical-chemical properties of the fly ash

The fly ash powder was dark gray, and its moisture content ranged from 0.97% to 2.54%. The composition of the fly ash was analyzed by XRF using the normalization method; the results are listed in Table 1. It can be observed that the fly ash primarily consisted of Si, K, Na, Ca, Fe, Al, Cl and S, which occupied approximately 87% of the total fly ash in mass. The Ca content was relatively high, which may have been caused by the lime spray during the acid gas control process during incineration. In addition, the Cl content in the fly ash was also high, which originates from the raw sludge and MSW. The higher Cl content will promote the enrichment of heavy metals in fly ash.

From Table 1, it can be observed that the Pb and Zn content in the fly ash were relatively high, whereas the Ni content was lower. This is primarily because Pb and Zn were release into the flue gas and adhered to the fly ash in the form of low-melting-point compounds, e.g., ZnCl_2_ and PbCl_2_, which were finally collected by the filter bags. The melting point of Ni is nearly 1726 K, and thus, the Ni will not volatilize; Ni primarily enters the bottom slag during incineration. Previous studies have shown that the nonvolatile elements with high boiling points are primarily concentrated in the bottom ash and the grate ash, whereas the volatile elements appeared in the fly ash^11^,^32^.

### Volatilization characteristics of heavy metals in pure fly ash

Thermal treatment time and reaction temperature are the key parameters to be considered in process development. Samples were heated at different temperatures (900 and 1000 °C) and at different residence times (60, 90, 120, 180, 240, 300 min) to study the volatilization of the four heavy metals. As shown in Fig. 2, under the same conditions, the *Ψ* values of the different metals differs significantly. During all of the conditions conducted without Cl addition, approximately 80–89% of the Pb, 48–56% of the Cd, 27–36% of the Zn and 6–24% of the Cu was volatilized. The volatility of the heavy metals in the sample and their removal followed the following sequence: Pb > Cd > Zn > Cu. It is hypothesized the reason why Cu exhibited the lowest volatilization is because of the low volatility of copper chlorides at 900 °C and 1000 °C. The boiling point of CuCl is 1450 °C, which is much higher than that of ZnCl_2_ (732 °C), CdCl_2_ (960 °C) and PbCl_2_ (950 °C). The low-boiling-point metals Pb and Cd have relatively high evaporating pressures, which mean they hardly react with the minerals to form stable compounds during a high temperature treatment and thus, easily become gaseous substances and have high evaporation rates.

For the same heavy metal (Fig. 2), it can also be observed that the variation curve of the evaporation rate against time at 900 °C differs only slightly from that at 1000 °C; both curves are smooth within the residence time from 60 to 300 min, which indicates the volatilization of heavy metals in the sample is only slightly affected by the reaction time, particularly for Pb and Cd. The results agree well with previous work, in which it has been proven that the evaporation rate of Cd and Pb is extremely high during thermal treatment due to their low melting and boiling points^11^,^27^.

At 900 °C, the *Ψ* of Pb increased from 80.40% to 89.62% when the residence time increased from 1 h to 5 h. After 1 h at 1000 °C, the *Ψ* of Pb was 82.87%. The same trend was observed at 900 °C, and the *Ψ* of Pb increased to 90.08% after 300 min of treatment. At 900 °C, more than 80% of the Pb was removed. However, during the subsequent thermal treatment, the effects of temperature and residence time on *Ψ* of Pb lessened.

The volatilization behavior of Cd was identical to that of Pb in the studied conditions. At 900 °C, the *Ψ* of Cd was 48.15% during the initial 1 h and reached 56.05% at a residence time of 5 h. While at 1000 °C, the *Ψ* of Cd increased slightly, from 49.26% to 57.97%. At temperatures of 900–1000 °C, the volatilization curve of Cd becomes flat as the residence time increases. Above 900 °C, the Cd contained in the fly ash volatilizes rapidly and is only slightly affected by increases in temperature and residence time.

The volatilization behaviors of Cu and Zn differed from that of Pb and Cd at the experimental conditions. At 900 °C, the *Ψ* of Cu was clearly low (6.04%); however, its growth after 240 min was larger than that of Cd, Pb and Zn. The *Ψ* of Zn increased rapidly during the initial 120 min and slowed down in the subsequent 180 min. At 1000 °C, the *Ψ* of Cu was high (19.73%) within the initial 90 min, whereas that of Zn varies only slightly from 28.58% to 37.1% during the entire thermal process. These results indicate that Cu is the most nonvolatile element, and its evaporation rate is lower than that of Pb and Cd in the selected metals. The bp(boiling point) of CuCl_2_ is 993 °C; however, in the temperature range of 900 to 1000 °C, the *Ψ* of Cu grows slowly (Fig. 2), i.e., the major compounds of Cu that appeared in the fly ash are likely are not in the form of chlorides but rather in forms of CuO or CuS^33^.

According to the volatilization behaviors, heavy metals can be classified into chalcophile or siderophile metals^34^. Cu is a chalcophile metal, which can easily vaporize above 900 °C. However, in this study however, the volatilization of Cu is not clear and had the lowest *Ψ* value. The melting points (boiling points) of PbO and PbCl_2_ are 886 °C(1472 °C) and 498 °C(954 °C), respectively^35^. For PbO, it is difficult to decompose but easy to volatilize at 900 °C–1000 °C, but above 950 °C, PbO began to volatilize dramatically. Pb may exist in MSS fly ash in the forms of both PbO and PbCl_2_, and thus, it clearly vaporizes rapidly from 900 °C to 1000 °C. For Cd, it appears in the MSS fly ash in the form of CdO and CdCl_2_, the melting point and boiling point of CdO are only 568 °C and 964 °C, respectively^36^. Thus, the volatilization of Cd and Pb exhibit similar trends at 900 °C and 1000 °C.

It can thus be inferred from the above results that in an oxidative atmosphere, from 900 °C to 1000 °C, the *Ψ* values of Pb and Cd are much greater than that of Cu and Zn. Pb and Cd exist primarily in the form of their chlorides in the fly ash, which have lower boiling points than their compounds in other forms. The metal chloride with a low boiling point is easy to volatilize. In the fly ash, a large part of Zn may be in the form of ZnO, which will react with SiO_2_ and Al_2_O_3_ during the process, which can be described equations (2,3)^37^,^38^.





During the stable compounds production, Zn_2_SiO_4_ and ZnAl_2_O_4_ are formed and can inhibit the evaporation of Zn, which is why the evaporation of Zn was lower than that of Pb and Cd. The low evaporation rate of Cu may be associated with its own nonvolatile performance. The above results agree well with the observations from previous studies^5^,^21^.

### Volatilization of heavy metals after the addition of chlorinating agents to fly ash

Effects of the amount and type of solid chlorinating agents on heavy metal removal were studied in this section. To be useful as a chlorinating agent, the chloride MCl_2_ must be able to react directly with metal oxides or release a chlorine-containing gas (Cl_2_ or HCl) when it react with oxygen or water according to the following general reactions, which are listed in equation (4,5)^29^.





The oxide MO should be chemically stable and have a low vapor pressure, such that the metal initially associated with the chlorinating agent will remain in the MSS fly ash and will not cause any environmental problem when the treated MSS fly ash is disposed of in a landfill. The chlorides in the forms of NaCl, CaCl_2_, MgCl_2_, FeCl_3_ and AlCl_3_ meet these requirements.

The MSS fly ash contains approximate 0.97–2.54% moisture, which is readily removed when the temperature is grater 100 °C. Several of the chlorinating agents contain not only moisture but also water crystallization. Both CaCl_2_ and MgCl_2_ may contain six H_2_O units per molecule. Upon heating, however, CaCl_2_ loses all water at temperatures greater than 200 °C^39^. Thus, chlorination by HCl, as described by Eq. (5), is unlikely to occur in a dry air system.

Figure 3 shows the effects of the different types and amounts of chlorinating agents on the removal of the four metals in the fly ash while holding the experimental conditions at 1000 °C for 1 h. It can be observed that after the chlorinating agents were added, the evaporation rate of the selected heavy metals Cu, Pb, Zn and Cd increased. Generally speaking, the degree of effectiveness of the chlorinating agents on heavy metal evaporation followed the following sequence: Cu > Zn > Cd > Pb. The *Ψ* values of Pb, Cd and Cu increased with the addition of 0.05 g of Cl into 5 g of ash regardless of the type of chlorinating agent. However, there was no significant improvement when more chlorinating agent was added. The addition of a chlorinating agent will not appreciably affect the vaporization of the existing metal chlorides. Thus, evidence from the high recovery of Pb, Cd and Cu with no additional chlorinating agent and from the recovery increase with the chlorinating agent addition suggests that an extremely large fraction of Pb, Cd and Cu is already in the form of chlorides. However, the strong dependence of the removal of Zn with the addition of more than 5% of chlorinating agents indicates that a significant fraction of Zn is in forms other than chlorides.

Lead can always be removed effectively from ash. The *Ψ* of Pb was 82.7% at 1000 °C for 60 min with no Cl added. After 1 wt.% of the chlorinating agent (FeCl_3_, AlCl_3_, MgCl_2_, CaCl_2_ and NaCl) was added to the fly ash, the *Ψ* of Pb increased from 82.7% to 94.40%, 95.69%, 94.52%, 95.28% and 91.58%, respectively. Moreover, when the proportion of the above chlorinating agents increased from 1% to 10%, the *Ψ* of Pb increased from 82.7% to 96.76%, 97.64%, 96.98%, 97.14% and 96.69%, respectively. The results indicate that chlorinating agents can enhance the *Ψ* of Pb, and *Ψ* increases as the chlorinating agent proportion increases. However, there is only a slight difference in the effects of the above five chlorinating agents on the volatilization of Pb. The enhancement for the *Ψ* of Pb with the added Cl was unclear because more than 80% of the Pb evaporated in the original fly ash.

Cadmium can be easily removed from ash-chloride mixtures. The *Ψ* of Cd was 49.16% at 1000 °C for 60 min without adding a chlorinating agent. With the addition of 1% of FeCl_3_, AlCl_3_, MgCl_2_, CaCl_2_ and NaCl, the *Ψ* of Cd increased from 49.16% to 65.61%, 74.01%, 70.56%, 70.44% and 71.52%, respectively. Moreover, when the proportion of the above chlorinating agents was increased from 1% to 10%, the *Ψ* of Cd reached 81.58%, 85.45%, 79.11%, 85.80% and 78.87%, respectively. The results indicate that chlorinating agents can enhance the evaporation rate of Cd, and the *Ψ* value of Cd increases as the chlorinating agent proportion increases. The enhancement of AlCl_3_ on the *Ψ* of Cd was the most significant, followed by the following in decreasing order: CaCl_2_ > FeCl_3_ > MgCl_2_ > NaCl.

Zinc exhibited a clear dependency on the type and amount of Cl added. The *Ψ* of Zn was 28.58% at 1000 °C for 60 min without an extra chlorinating agent added. With an addition of 1% of FeCl_3_, AlCl_3_, MgCl_2_, CaCl_2_ and NaCl, the *Ψ* of Zn increased from 28.58% to 33.22%, 34.47%, 50.05%, 67.74% and 41.83%, respectively. Moreover, when the proportion of the above chlorinating agents increased from 1% to 10%, the *Ψ* value of Zn reached 76.46%, 80.21%, 90.75%, 85.93% and 70.10%, respectively. The improvement of the above five chlorinating agents on the volatilization of Zn followed the following sequence: MgCl_2_ > CaCl_2_ > FeCl_3_ > AlCl_3_ > NaCl.

At 1000 °C for 60 min without extra Cl added, 13.28% of Cu can be released. With an addition of 1% of FeCl_3_, AlCl_3_, MgCl_2_, CaCl_2_ and NaCl, the Cu increased from 13.28% to 60.66%, 60.95%, 66.21%, 49.74% and 52.26%, respectively. Moreover, when the proportion of the above chlorinating agents increased from 1% to 10%, the evaporation rate of Cu reached 92.46%, 90.35%, 86.84%, 87.86% and 54.90%, respectively. This result indicates that the chlorinating agents can greatly enhance the evaporation rate of Cu, and the evaporation rate of Cu increases as the chlorinating agent proportion increases (except for NaCl). With an increase of 0–15% NaCl, the evaporation rate of Cu first increased (0–5% of NaCl) and then decreased (5–15%). The improvement of the five chlorinating agents on the volatilization of Cu followed the following sequence: FeCl_3_ > AlCl_3_ > MgCl_2_ > CaCl_2_ > NaCl.

The equilibrium partial pressures of the chloride decreased according to the sequence AlCl_3_, MgCl_2_, FeCl_3_,CaCl_2_, and NaCl in the temperature range of 600–1200 °C^21^. When chlorination is a necessary step for metal removal, such as the removal of Zn in this case, there should be a certain dependence of *Ψ* on the type of chlorinating agent. Figure 3 shows that NaCl, FeCl_3_ and AlCl_3_ were less effective at 1000 °C than MgCl_2_ and CaCl_2_ in the removal of Zn. In the air, NaCl has less of a tendency to supply chlorine than other chlorinating agents. Another consideration is the volatility of the chlorinating agent itself. The vapor pressure of NaCl is two orders of magnitude greater than that of CaCl_2_ at 1000 °C. As a result, it is easier for NaCl to evaporate without reacting with oxygen or metal oxides and to end up with the volatile matter. In other words, less NaCl will be available as a chlorinating agent. An analysis of the sodium content of the condensed matter revealed that 62% of the sodium salt ended up with volatile matter after 3 h of heating at 1000 °C compared with less than 1% of Ca, Mg and Fe salts^21^. The ineffectiveness of AlCl_3_ is due to its high tendency to release chlorine at relatively low temperatures, at which the rate of chlorination of Zn is not significant. In fact, AlCl_3_ is the only chlorinating agent tested that has an extremely high equilibrium partial pressure of chloride at low temperatures. However, to remove Zn via chlorination, the temperature must be greater than 600 °C^21^. Thus, AlCl_3_ may have released chlorine before the reaction with zinc oxide could have occurred According to Fig. 3, there was no significant difference between the removal of heavy metals using MgCl_2_, CaCl_2_ or FeCl_3_. When these chlorides are used, the partial pressure of chloride in the system remained the same. The reaction between the oxygen and chlorinating agent may be controlled by the oxygen partial pressure in the air, which is close to constant in an open system, such as that used in this experiment.

### SEM-EDS and XRD analysis

The SEM image of the fly ash after thermal treatment at different temperatures is shown in Fig. 4. It can be observed that with increasing temperature, the fly ash particles become larger, harder and denser. The loose and accumulated particles gradually become massive, and the pore space between the particles also reduces, which inhibits the evaporation of heavy metals at high temperatures.

Figure 5 shows the EDS image of the fly ash after being treated at different temperatures. It can be observed that with an increase in temperature, the content of the major elements, such as Ca, Fe, Al and Si, in the MSS fly ash changes only slightly, whereas that of certain volatile elements, including Cl, C and S, and semi-volatile heavy metals, such as Pb, Cd and Zn, reduces dramatically. For example, when the temperature was raised from 900 °C to 1000 °C with a residence time of 1.5 h, the contents of Na, Mg, Al, Si, S, Cl, K, Ca, Fe and Pb decreased from 1.47%, 1.23%, 4.04%, 7.38%, 2.62%, 0.72%, 0.88%, 12.02%, 11.47% and 0.44% to 1.13%, 1.15%, 3.71%, 7.35%, 1.36%, 0.06%, 0.79%, 10.58%, 9.56% and 0.1%, respectively.

The SEM images of the fly ash treated at 1000 °C for 60 min with and without 10% chlorinating agents are shown in Fig. 6. It can be observed that without the chlorinating agent addition, the MSS fly ash particles melt and remain close together after thermal treatment; the particles are dense, massive and contain small voids (see Fig. 7a). When different chlorinating agents are added to the MSS fly ash, the morphology of the heated fly ash changed significantly. The fly ash particles are presented as spherical, speculate, petaloid and massive shapes. Large spaces exist between particles; the particles are loose and smooth, which are all qualities that are beneficial to heavy metal evaporation. When the proportion of the chlorinating agents increased from 1% to 10%, most of the Cl vaporized after reacting with the heavy metals. Figure 7 shows the EDS images of the fly ash at 1000 °C with an addition of 10% chlorinating agents. It can see that from Fig. 8 that it is difficult for NaCl to react with the heavy metals to form the corresponding chlorides. Thus, NaCl has only a slight little effect on the *Ψ* of the heavy metals. The two chlorinating agents, FeCl_3_ and AlCl_3_, have a stronger improvement effect on the evaporation rate of heavy metals than that of NaCl.

Figure 9 shows the XRD pattern of the pure MSS fly ash sample. Calcium-bearing compounds were rich in pure fly ash. The major calcium crystalline phase (CaSO_4_, CaCO_3_, CaO and CaAl_2_SiO_6_) and the chloride compound (KCl, NaCl, CaCl_2_, Ca(OH)Cl) were identified. The compounds of CaCl_2_·2H_2_O and Ca(OH)Cl are both chlorinated products of the reaction between Ca(OH)_2_ and HCl during the acidic gas removal process by adding the lime in the spray-dryer system according to equations (6–8)^40^:







The reaction between Ca(OH)_2_ and HCl most likely forms Ca(OH)Cl.

XRD patterns of the chlorinated ashes obtained after adding chlorinating agents are presented in Fig. 9. It can be observed that with the chlorinating agents addition, more complex aluminosilicates were newly formed due to the increased temperature, e.g., anorthite (CaAl_2_Si_2_O_8_), merwinite (Ca_3_Mg(SiO_4_)_2_), and aluminosilicate (Ca_3_Al_6_Si_2_O_16_). However, the intensity of KCl, NaCl, CaCl_2_ and Ca(OH)Cl decreased significantly at 1000 ^°^C, which indicates that these minerals were completely vaporized or decomposed. The mineralogical forms of the heavy metals could not be identified because of their amorphous structure and low concentration.

The four heavy metals can be removed to a certain extent from the MSS fly ash with the addition of different chlorinating agents. After the chlorinating agents were added to the MSS fly ash, the forms of Cu, Zn and Pb were extremely likely to change and exist in their chlorides forms during the thermal treatment process, whereas Cd appeared in the form of its oxides and chlorides, which would increase its evaporation rate. Additionally, from Fig. 8, it can be observed that the presence of Cl can enhance the volatilization of metals compared with the vapor pressures of the heavy metals and their chlorides^41^. Therefore, the heavy metal compounds or other forms in the fly ash should be transformed into the corresponding chlorides to improve the recovery or removal rate of the selected metals. The above results show that adding chlorinating agents is an effective method; however, anti-corrosion measures should be concurrently taken for the devices.

### Reaction mechanism for heavy metal removal

The addition of chlorinating agent can enhance the removal of metal by a mechanism other than only supplying chlorine. Using CaCl_2_ as an example, the enhancement of chlorinating agents on the *Ψ* of heavy metals is as follows. CaCl_2_ reacts with O_2_ in the air, and Cl_2_ is generated during this process. Then, Cl_2_ reacts with the heavy metal oxide (MO) and transforms into low-boiling-point metal chlorides. The detailed chemical process is expressed by equations (9–11)^21^.





The above two processes can be combined and simplified as the following:



Table 2 lists the variations of the Gibbs free energy (Δ*G*) of several reactions between heavy metal oxides and Cl at 1050 °C, in which Δ*G* < 0 indicates that the reaction goes in the positive direction.

During the thermal treatment, chlorinating agents either react directly with heavy metal oxides or form HCl or Cl_2_ by reacting with H_2_O or O_2_. HCl and Cl_2_ subsequently chlorinate heavy metal oxides (indirect chlorination). For direct reaction, evaporation (or at least melting) of chloride is necessary because the ash–chloride mixture is not perfectly homogenized. According to the equilibrium calculations^42^, NaCl does not (or hardly) react with H_2_O and O_2_, neither in a pure system nor in systems containing heavy metal oxides. Due to the NaCl with high vapor pressure, it evaporates in high quantities without reacting sufficiency^21^; here, at 1000 °C, 10% of NaCl was already in gaseous forms in this study. For CaCl_2_, equilibrium calculations reveal that heavy metal volatilization can principally follow the route of both direct and indirect chlorination, leading to approximately the same fractions of heavy metals volatilized. The reaction of CaCl_2_ with H_2_O and O_2_ is thermodynamically and also kinetically favored compared with evaporation and the maximum amount of heavy metals evaporable is much greater with Cl_2_ or HCl^42^,^43^,^44^. For MgCl_2_, indirect chlorination is the most probable pathway for heavy metal removal because the release of HCl or Cl_2_ is thermodynamically more stable than that of salt^29^.

## Conclusions

- (1) During the pure MSS fly ash thermal treatment, approximately 80 to 89% of Pb, 48 to 56% of Cd, 27 to 36% of Zn and 6 to 24% of Cu were volatilized. During this process, temperature was an important parameter and had significant influence on the volatilization of heavy metals, whereas residence time had the weakest effect, particularly for Pb and Cd, which easily volatize.
- (2) Chlorinating agents exhibited an apparent promoting effect on heavy metals removal, particularly for the mid-volatile metals, Cu and Zn. With an addition of 10 wt% chlorinating agents, more than 96% of Pb, 78% of Cd, 76% of Zn (except NaCl) and 86% of Cu (except NaCl) can be removed from MSS ash. With an increase in Cl proportion, the evaporation rate of the heavy metals increased; however, the effect clearly varied. The NaCl had the weakest enhancement effect on the evaporation rate of Cd, Zn and Cu.
- (3) The best choice of chlorinating agents is in the order of MgCl_2_ > CaCl_2_ > FeCl_3_ > AlCl_3_ > NaCl due to the metal removals (particularly Zn) and the low amount of remaining chlorine, which favors treated ash for further resource use or disposal.

## Additional Information

**How to cite this article**: Liu, J. Y. *et al.* Heavy metal removal from MSS fly ash by thermal and chlorination treatments. *Sci. Rep.* **5**, 17270; doi: 10.1038/srep17270 (2015).

## Figures and Tables

**Figure 1:** Experimental apparatus of quartz tube simulation combustion reactor.

**Figure 2:** Volatilization characteristics of heavy metals in fly ash without chlorination agent at (**a**) 900 °C, (**b**) 1000 °C.

**Figure 3:** Effects of amount and type of chlorination agents on evaporation rate of heavy metals in fly ash (holding at 1000 °C for 60 min).

**Figure 4:** SEM photograph of fly ash after incineration at (**a**) 800 °C (**b**) 900 °C (**c**) 1000 °C (**d**) 1100 °C for 1.5 hours.

**Figure 5:** EDS photographs of fly ash after incineration at (**a**) 800 °C (**b**) 900 °C (**c**) 1000 °C (**d**) 1100 °C for 1.5 hour.

**Figure 6:** SEM photographs of fly ash with (**a**) 0% chlorination agent (**b**) 10% CaCl_2_ (**c**) 10% MgCl_2_ (**d**) 10% NaCl (e) 10% FeCl_3_ and (f) 10% AlCl_3_ after incineration at 1000 °C for 60 min.

**Figure 7:** EDS photographs of fly ash with (**a**) 0% chlorination agent (**b**) 10% CaCl_2_ (**c**) 10% MgCl_2_ (**d**) 10% FeCl_3_ (**e**) 10% AlCl_3_ and (**f**) 10% NaCl after incineration at 1000 °C for 60 min.

**Figure 8:** Vapour pressures of (**a**) heavy metals and (**b**) their chlorides.

**Figure 9:** XRD of MSS fly ash before and after calcination with the addition of chlorinating agents. 1. CaSO_4_; 2. CaCO_3_; 3.NaCl; 4. KCl; 5. Ca_2_Al_2_SiO_7_; 6. Ca_2_(PO_4_)_3_; 7. CaO; 8. SiO_2_; 9. CaAl_2_SiO_6_; 10. CaClOH; ⑪. CaAl_2_Si_2_O_8_; ⑫. Ca_3_Mg(SiO_4_)_2_; ⑬. NaCa_4_Al_3_O_9_; ⑭. Ca_3_Al_6_Si_2_O_16_; ⑮Al_2_O_3_; ⑯NaCa_4_Al_3_O_9_; ⑰CaSiO_3_; ⑱Fe_2_O_3_; ⑲nFe_2_Al_4_Si_5_O_18._

**Table 1:** Chemical composition and heavy metal content in fly ash.

Chemical composition of fly ash	Content*(%)*
Al_2_O_3_	8.81
CaO	13.13
Fe_2_O_3_	12.39
K_2_O	4.97
MgO	1.94
MnO	0.12
Na_2_O	3.75
P_2_O_5_	1.59
SiO_2_	23.48
TiO_2_	0.62
Cl	11.25
SO_3_	8.74
**Heavy metal contents in fly ash**	**(mg/kg)**
Cu	857
Pb	1359
Cd	29.4
Cr	612
Ni	187
Mn	1524
Zn	3288

**Table 2:** Gibbs free energy change of reaction between heavy metal oxide and Cl_2_ at 1050 °C.

Reaction equation	Δ*G*/kJ·mol^−1^
	−160
	−88
	−112
	−180
